The article "Cytotoxic effect of a new 1,3,4-thiadiazolium mesoionic compound (MI-D) on cell lines of human melanoma" was published in 2004. Journal: Br J Cancer.

# Cytotoxic effect of a new 1,3,4-thiadiazolium mesoionic compound (MI-D) on cell lines of human melanoma

**DOI:** 10.1038/sj.bjc.6601946

**Published:** 2004-06-15

**Authors:** A Senff-Ribeiro, A Echevarria, E F Silva, C R C Franco, S S Veiga, M B M Oliveira

**Affiliations:** 1 Department of Biochemistry and Molecular Biology, Federal University of Paraná, Curitiba, PR, Brazil; 2 Department of Chemistry, Rural Federal University of Rio de Janeiro, Rio de Janeiro, RJ, Brazil; 3 Department of Cellular Biology, Federal University of Paraná, Curitiba, PR, Brazil

**Keywords:** mesoionic compounds, MI-D, antimelanoma activity, human melanoma cell lines

## Abstract

The structural characteristics of mesoionic compounds, which contain distinct regions of positive and negative charges associated with a poly-heteroatomic system, enable them to cross cellular membranes and interact strongly with biomolecules. Potential biological applications have been described for mesoionic compounds. 1,3,4-Thiadiazolium mesoionic compound (MI-D), a new mesoionic compound, has been demonstrated to be extremely cytotoxic to B16-F10 murine melanoma cells when compared to fotemustine and dacarbazine, drugs of reference in melanoma treatment protocols, describing inhibition of tumours grown *in vitro* and *in vivo*. We now evaluate the effects of mesoionic compound MI-D on different human melanoma cell lines. The drug decreased the viability and proliferation of MEL-85, SK-MEL, A2058 and MEWO cell lines *in vitro*, showing a considerable cytotoxic activity on these human cells. Adhesion of MEL-85 cells was evaluated in the presence of the drug using different extracellular matrix (ECM) constituents. MI-D decreased MEL-85 adhesion to laminin, fibronectin and matrigel. The morphology and actin cytoskeleton organisation of MEL-85 cells were also modified on MI-D treatment. These results on human melanoma cell lines indicate that MI-D is a very encouraging drug against melanoma, a tumour that is extremely resistant to chemotherapy.

Compounds of the mesoionic class have interesting structural features provided by their betaine-like character. They consist of a five-membered heterocyclic ring associated with a sextet of p and *π* electrons, supporting a partial positive charge in the heterocyclic ring, which is counterbalanced by a formal negative charge on the atom of the *α*-side chain (Ollis and Ramsden, 1976; Newton and Ramsden, 1982; Cheung *et al*, 1992). The association of these characteristics suggests a high probability of strong interactions with biomolecules such as DNA and/or proteins. Although mesoionic compounds are internally charged, they are neutral overall, and can therefore cross biological membranes *in vivo* (Kier and Roche, 1967).

The article "Cytotoxic effect of a new 1,3,4-thiadiazolium mesoionic compound (MI-D) on cell lines of human melanoma" was published in 2004. Journal: Br J Cancer.

All the different classes of mesoionic compounds (sydnones, sydnonimines, isosydnones and 1,3,4-thiadiazoles) have received considerable attention and have been extensively studied because of their unique structures, reaction behaviour, biological activities and possible pharmaceutical use (Moustafa and Eisa, 1991; Corell *et al*, 1994; Rehse *et al*, 1995; Satyanarayana and Rao, 1995). These include anti-inflammatory, analgesic, antibacterial, antifungal and antitumour activities (Badachikar *et al*, 1986; Shinzato *et al*, 1989; Moustafa and Eisa, 1991; Grynberg *et al*, 1992; Montanari *et al*, 1992; Satyanarayana and Rao, 1995; Grynberg *et al*, 1997; Senff-Ribeiro *et al*, 2003, 2004). Potent antiplatelet, fibrinolytic, thrombolytic and broncholytic effects (Corell *et al*, 1994; Kankaanranta *et al*, 1996), and effects on the cardiovascular system (Majid *et al*, 1980; Rudolph and Derschinger, 1991; Rehse and Konig, 1995; Rehse *et al*, 1995) have also been described for mesoionic compounds. Some effects described for these compounds are intimately related to the presence of specific substituent groups on the ring (Corell *et al*, 1994; Satyanarayana and Rao, 1995; Kankaanranta *et al*, 1996; Grynberg *et al*, 1997), or to the ability to release nitric oxide from their molecular structures (Hogg *et al*, 1992).

A new mesoionic compound, 4-phenyl-5-(4-nitrocinnamoyl)-1,3,4-thiadiazolium-2-phenylamine chloride (MI-D) was synthesised by Grynberg *et al* (1997) (Figure 1

**Figure 1:** Chemical structure of 4-phenyl-5-(4-nitrocinnamoyl)-1,3,4-thiadiazolium-2-phenylamine chloride (MI-D).

), for which it was shown the enhancement of the survival of Ehrlich carcinoma and Sarcoma-180 tumour-bearing mice, preventing tumour growth, with no significant concomitant alterations in the haematological parameters of tested animals, at a dose of 25 mg kg^−1^ (57 *μ*mol kg^−1^).

MI-D was shown to be able to inhibit the respiratory chain between complexes II and III, collapse the transmembrane potential, and stimulate ATPase activity in intact mitochondria (Cadena *et al*, 1998). Alterations were also reported in membrane permeability and fluidity, which are related to its effect on the energy-linked functions of mitochondria (Cadena *et al*, 2002).

Recent studies in our laboratory evaluating a series of 1,3,4-thiadiazolium mesoionics showed that MI-D, which has an NO_2_ substituent on the cinnamoyl ring, was the most effective against the melanoma murine model B16-F10 (Senff-Ribeiro *et al*, 2004). Compared with two other antineoplastic agents (fotemustine and dacarbazine), it was effective against the murine model both *in vitro* and *in vivo*, under the same experimental conditions and with the same molar concentrations (Senff-Ribeiro *et al*, 2003).

The article "Cytotoxic effect of a new 1,3,4-thiadiazolium mesoionic compound (MI-D) on cell lines of human melanoma" was published in 2004. Journal: Br J Cancer.

Although antitumour effects against Ehrlich and Sarcoma-180 tumour models, and even against the aggressive melanoma murine model B16-F10, have already been demonstrated for MI-D (Grynberg *et al*, 1997; Senff-Ribeiro *et al*, 2003, 2004), it has not been tested against human melanoma cell lines.

We now study the effects of MI-D on four established human melanoma cell lines: MEL-85, SK-MEL, A2058 and MEWO. The *in vitro* viabilities and proliferations of these cell lines in the presence of MI-D were evaluated. In order to obtain further insights concerning MI-D's anti-melanoma activity, cell features of adhesion, morphology and actin cytoskeleton organisation, which are deeply related to the development and establishment of tumours, were also subjects studied using the MEL-85 cell line.

## MATERIALS AND METHODS

### Materials

MI-D (4-phenyl-5-(4-nitro-cinnamoyl)-1,3,4-thiadiazolium-2-phenylamine chloride) was synthesised in the Department of Chemistry of the Rural Federal University of Rio de Janeiro, Brazil, as described elsewhere (Grynberg *et al*, 1997). Its structure was confirmed by ^1^H- and ^13^C-NMR spectroscopy and mass spectrometry. Dulbecco's modified Eagle's medium (DMEM), RPMI1640 medium and fetal bovine serum (FBS) were obtained from Cultilab (Campinas, Brazil); penicillin and gentamycin were both purchased from GIBCO (Bethesda, USA). Paraformaldehyde (20%, aqueous solution) was from EMS (Electron Microscopy Sciences, Washington, USA). Phalloidin labelled with FITC was from Molecular Probes (Eugene, USA) and the aqueous mounting medium, Fluormount-G® from EMS (Washington, USA). Trypan blue, MTT, crystal violet and glycine were obtained from Sigma Aldrich (St Louis, USA). DMSO was from Merck. All other reagents were commercial products of the highest available purity grade.

### Drug solutions

MI-D was dissolved in dimethylsulphoxide (DMSO) for its experimental use. In order to minimise solvent interference, several stock solutions of MI-D were prepared so that at the desired final concentrations of MI-D in the assays, the amounts of DMSO were identical and equal to 0.12%.

### Cell lines and culture conditions

Human melanoma cell lines used in this study were kindly provided by the Ludwig Institute for Cancer Research (São Paulo, Brazil). Cells were maintained in liquid nitrogen with a low number of passages. After thawing, the cells were grown in monolayer cultures in the appropriate media containing penicillin (100 U ml^−1^) and gentamicin (50 *μ*g ml^−1^). MEL-85 and MEWO cells were cultured in RPMI containing 10% FBS, SK-MEL cells in RPMI containing 15% FBS and A2058 cells in DMEM containing 10% FBS. The cultures were kept at 37°C under a humidified atmosphere plus 5% CO_2_. Release of cells was performed by a treatment for a few minutes with a 2 mM solution of ethylenediaminetetraacetic acid (EDTA) in phosphate-buffered saline (PBS). After being counted, cells were then resuspended in an adequate volume of the respective medium supplemented with FBS and again plated in the presence or absence of MI-D.

The article "Cytotoxic effect of a new 1,3,4-thiadiazolium mesoionic compound (MI-D) on cell lines of human melanoma" was published in 2004. Journal: Br J Cancer.

### Cell viability assay

Viability assays were carried out on 24-well plates (TPP, Trasadingen, Switzerland). Human melanoma cells (5 × 10^5^ cells well^−1^) were plated and allowed to adhere and grown for 20 h before incubation with the drug. MI-D was added in varying concentrations up to 75 *μ*M. At each determined interval (24 and 48 h), supernatants and cells were harvested, centrifuged, washed with PBS and the viability was measured by the Trypan blue-exclusion assay (Phillips, 1973). Briefly, Trypan blue (0.4% in PBS, pH 7.4) was added to the cell suspension and the number of viable (unstained) and nonviable (stained) cells was counted using a Neubauer Chamber. For control experiments, the appropriate medium contained adequate amounts of vehicle (0.12% of DMSO). Cell viability of controls was normalised to 100%.

### Cell proliferation assay

Human melanoma cells (6 × 10^3^ cells well^−1^) were grown for 16 h on 96-well plates (TPP) containing an appropriate medium supplemented with an adequate amount of FBS. The medium was then replaced by a serum-free one. After 24 h, this was replaced with the respective medium containing the usual concentrations of FBS plus MI-D, at different concentrations (2.5–25 *μ*M) in quadruplicate. Controls consisted of the respective medium alone or in the presence of 0.12% DMSO, which was the MI-D solvent. After 24, 48 and 72 h the number of cells in each well was determined using the MTT method (Mosmann, 1983). MTT [3-(4,5-dimethylthiazol-2-yl)-2,5-diphenyl tetrazolium bromide] was dissolved in Hanks’ balanced saline solution (HBSS) at 5 mg ml^−1^. At the above intervals, 20 *μ*l of the MTT solution were added to each well and the plates were incubated at 37°C for 3 h. The MTT solution was removed and DMSO was added and mixed thoroughly to dissolve the dark-blue crystals. The plates were then read using a Microelisa Reader (Bio-Rad, Madison, USA) at 550 nm for sample and 655 nm for reference. Results are expressed as the cell number, which was determined using a standard curve of cells against absorbance.

### Cell adhesion assay

Native fibronectin was purified from fresh human plasma according to the procedure of Engvall and Ruoslahti (1977). Laminin and matrigel, a reconstituted basement membrane, were purified from a Engelbreth–Holm–Swarm (EHS) tumour as described by Paulsson *et al* (1987) and Kleinman *et al* (1986), respectively. The presence and purity of proteins were assessed by both an electrophoretic analysis on sodium dodecyl sulphate–polyacrylamide gel electrophoresis (SDS–PAGE) and Western blot. Adhesion assays were performed as described by Saiki *et al* (1989) with some modifications. Briefly, MEL-85 cells (4 × 10^4^) with or without MI-D (0.5, 1.0, 2.5 and 5.0 *μ*M) were added to microculture wells (96-well plates, TPP) precoated with fibronectin, laminin or matrigel (10 *μ*g ml^−1^) and blocked with bovine serum albumin (BSA) 1%. The cultures were incubated at 37°C for 2 h. The wells were washed twice with warm PBS to remove unattached cells, and then the attached cells were fixed with methanol and stained with 0.8% crystal violet dissolved in 20% ethanol. After extensive washing with PBS, the dye was eluted with 50% ethanol in 0.05 M sodium citrate and the absorbance was measured at 550 nm using a MicroElisa Reader (BioRad). At the end of the experiment, the plates were photographed (Leica-MPS30) using an inverted microscope (Leica-DMIL). The control contained the same amount of DMSO as the tested wells (0.12% of DMSO) and its cellular adhesion was normalised to 100%.

The article "Cytotoxic effect of a new 1,3,4-thiadiazolium mesoionic compound (MI-D) on cell lines of human melanoma" was published in 2004. Journal: Br J Cancer.

### Cell morphology analysis

MEL-85 cells were cultured on glass coverslides for 16 h at 37°C under a humidified atmosphere plus 5% CO_2_. Cells were treated with 25 and 50 *μ*M MI-D for 2 h. After treatment, they were washed twice with PBS and fixed with 2% paraformaldehyde in PBS for 30 min at 4°C. For the control, the appropriate medium contained adequate amounts of vehicle (0.12% of DMSO). Coverslides were stained by Giemsa and studied by bright-field microscopy (Olympus BX40). Images were acquired (× 400) in grayscale using a software Image-Plus 4.0 version (Media Cybernetics, Silver Spring, USA). A morphometric analysis was performed using an ImageTool software 3.00 version (University of Texas Health Science Center in San Antonio, USA). Cell features, such as area, elongation and roundness of about 400 cells were analysed. For analysis, the area of the object, measured as the number of pixels in the polygon was converted to percent. Elongation was measured as the ratio of the length of the major axis to the length of the minor axis. The result was a value of between 0 and 1 that was converted to % for analysis to obtain an analytical value. Roundness was computed as: (4*π* × area)/perimeter^2^. The result gave a value of between 0 and 1 that was converted to % for analysis.

The article "Cytotoxic effect of a new 1,3,4-thiadiazolium mesoionic compound (MI-D) on cell lines of human melanoma" was published in 2004. Journal: Br J Cancer.

### Immunofluorescence microscopy

MEL-85 cells (5 × 10^4^) were plated on glass coverslides (13 mm diameter), which were prepared for confocal immunofluorescence microscopy. After 16 h, MEL-85 cells were incubated with 50 *μ*M MI-D for 2 h at 37°C under a humidified atmosphere plus 5% CO_2_. In the control, the appropriate medium contained adequate amounts of vehicle (0.12% of DMSO). Cells were washed twice with PBS and fixed with 2% paraformaldehyde in PBS for 30 min at 4°C. Cells on coverslides were incubated with 0.1 M glycine for 3 min, washed with PBS and then blocked with PBS containing 1% BSA for 30 min at room temperature (25°C). After washing thrice with PBS, coverslides were incubated with phalloidine conjugated with fluorescein isothiocyanate (FITC) (Molecular Probes) diluted in PBS (1 : 200) for 20 min. After washing with PBS (10 ×) and once in water, slides were mounted with Fluormont-G®. Cells were observed using a confocal fluorescence microscope (Confocal Radiance 2100, Bio-Rad) coupled to a Nikon Eclipse 800 with plan apochromatic objectives (Science and Technologies Group Instruments Division, Melville, USA). Images were acquired (× 600) using Radiance 2100 (Bio-Rad).

### Statistical analysis

Statistical analysis of data were carried out using analysis of variance (ANOVA) and the Tukey test for average comparison. Mean±s.d. values were used. Significance was defined as *P*<0.05.

## RESULTS

### Effect of MI-D on cell viability

Figure 2

**Figure 2:** Effects of MI-D on the viability of different human melanoma cell lines. (**A**) Effects of MI-D on MEL-85 cells. (**B**) Effects of MI-D on SK-MEL cells. (**C**) Effects of MI-D on A2058 cells. (**D**) Effects of MI-D on MEWO cells. The viability of melanoma cells was measured at indicated intervals and concentrations of MI-D using the trypan blue-exclusion assay (*n*=4). Values given are the mean±s.d. ^*^P<0.001.

shows the effect of the mesoionic compound on the viability of human melanoma cell lines evaluated 24 and 48 h after treatment with different concentrations of MI-D (2.5–75 *μ*M). Time- and dose-dependent effects were shown by MI-D on the four cell lines studied.

The viability of MEL-85 cells was reduced to 56% after a 24 h treatment with 10 *μ*M MI-D (Figure 2A). At this time of incubation, 75 *μ*M MI-D diminished the viability by ∼82%. When a treatment of 48 h was used, the maximum cytotoxic effect (100%) was reached starting from 50 *μ*M. A measure of 5 *μ*M MI-D reduced the number of viable cells to 27% after 48 h incubation.

SK-MEL cells also had their viability diminished by MI-D treatment (Figure 2B). After 24 h, 25 *μ*M MI-D reduced the viability to ∼30% and at 50 *μ*M to 17%. When the concentration was raised to 75 *μ*M, there were no viable cells after 24 h incubation. A volume of 10 *μ*M MI-D reduced the viability to 30% after 48 h. At this time, there was more than 90% of cell death using 50 *μ*M MI-D.

The article "Cytotoxic effect of a new 1,3,4-thiadiazolium mesoionic compound (MI-D) on cell lines of human melanoma" was published in 2004. Journal: Br J Cancer.

The viability of A2058 cells was decreased to ∼30% when the concentration of MI-D was 10 *μ*M and the incubation time was 24 h (Figure 2C). At this time, the concentrations of 25 and 50 *μ*M reduced the number of viable cells to 12 and 7%, respectively. When a 48 h incubation was assayed, 10 *μ*M MI-D reduced the viability to 20% and 25 *μ*M almost gave a maximum cytotoxic effect (97%). At this time, all A2058 cells were dead when the concentration of MI-D was 50 *μ*M.

MEWO cells were also very sensitive to the toxic effects of MI-D (Figure 2D). After 24 h, MI-D at 10 and 25 *μ*M concentrations, diminished the viability to 23 and 8%, respectively. Increasing the drug concentration to 75 *μ*M resulted in only ∼1% of viable cells after 24 h. When a 48 h treatment was performed, 10 *μ*M MI-D reduced the number of viable cells to 13% while 50 *μ*M gave rise to ∼100% cell death.

### Effect of MI-D on cell growth

Evaluation of the effect of MI-D on the growth of human melanoma cell lines was performed using a growth–time kinetic study of up to 72 h (Figure 3

**Figure 3:** Effects of MI-D on the proliferation of human melanoma cell lines. (**A**) Effects of MI-D on MEL-85 cells. (**B**) Effects of MI-D on SK-MEL cells. (**C**) Effects of MI-D on A2058 cells. (**D**) Effects of MI-D on MEWO cells. The proliferation rates were measured using the MTT method at the times indicated and at subcytotoxic (2.5 *μ*M) and cytotoxic (5–25 *μ*M) concentrations (*n*=3). Values given are the mean±s.d. ^*^P<0.01 ^**^P<0.001.

). Proliferation of all melanoma cell lines was greatly inhibited by MI-D, even when subcytotoxic concentrations (1–2.5 *μ*M) were tested.

MEL-85 cells (Figure 3A) treated with 5 *μ*M MI-D gave a 50% reduction of cell growth during the 72 h experiment. At a concentration of 10 *μ*M, the proliferation of MEL-85 cells was completely inhibited.

No growth of SK-MEL cells (Figure 3B) was observed when 5 *μ*M MI-D was used. After 24 h, 1 and 2.5 *μ*M MI-D reduced the number of cells to ∼65 and ∼55%, respectively.

A2058 cells (Figure 3C) had their growth reduced to 55–61% when the concentration was 2.5 *μ*M. When MI-D was used at 5 *μ*M, there was no increase in cell number up to 48 h. However, at 72 h there was a recovery and the number of cells increased, being 46% of the control.

The proliferation of MEWO cells was inhibited by MI-D (Figure 3D). At a low MI-D dose (2.5 *μ*M) a decrease of cell number of a quarter after 48 and 72 h was observed. The concentration of 5 *μ*M allowed cell growth up to 24 h, but after there was no increase in cell number up to 72 h. In all, 10 *μ*M MI-D did not allow MEWO growth. It must be pointed out that all cell lines, when exposed to MI-D at 10 *μ*M or more, did not grow and extensive cell death was observed, confirming the previous data appearing in Figure 2.

The article "Cytotoxic effect of a new 1,3,4-thiadiazolium mesoionic compound (MI-D) on cell lines of human melanoma" was published in 2004. Journal: Br J Cancer.

### Effect of MI-D on MEL-85 adhesion to laminin, fibronectin and matrigel

Figure 4

**Figure 4:** Effects of MI-D on the adhesion of MEL-85 human melanoma cell to ECM constituents. (**A**) MEL-85 adhesion to laminin. (**B**) MEL-85 adhesion to fibronectin. (**C**) MEL-85 adhesion to matrigel. (**D**) Micrographs of MEL-85 cells adhered to fibronectin. (1) Control cells, (2) cells treated with 2.5 *μ*M MI-D, (3) cells treated with 5 *μ*M MI-D. MEL-85 cells (4 × 10^4^) were added to microculture wells precoated with ECM constituents in the presence of indicated concentrations of MI-D. After a 2 h incubation, nonadherent cells were washed and adherent cells were fixed and stained with 0.8% (p v^−1^) crystal violet containing 20% methanol. After extensive washing, the stained cells were lysed with 50% ethanol in 0.05 M sodium citrate and the absorbance was measured at 550 nm. ^**^P<0.01 and ^***^P<0.001.

shows the effects of MI-D on MEL-85 adhesion to extracellular matrix (ECM) constituents, such as laminin, fibronectin and matrigel. Although there were apparent decreases on cell adhesion when 0.5 and 1 *μ*M of MI-D were used, the values were not statistically different from those of the controls. Higher concentrations of MI-D significantly inhibited MEL-85 adhesion to ECM molecules in a concentration-dependent manner. Adhesion to laminin and fibronectin was decreased to 70 and 55% by 2.5 and 5 *μ*M of MI-D, respectively, after 2 h exposure (Figures 4A and B). At 5 *μ*M, MI-D diminished MEL-85 adhesion to laminin to ∼65% (Figure 4A) and to fibronectin and matrigel to 34 and 71%, respectively (Figure 4B and C). The micrographs of the adhesion on fibronectin (Figure 4D) show that MI-D not only reduced the number of cells adhering to fibronectin, but also altered the morphology of MEL-85 cells, which shrinked and became round. These changes were also observed when cells were assayed for their adhesion on laminin and matrigel (data not shown).

### Effect of MI-D on MEL-85 morphology

Figure 5

**Figure 5:** Effects of MI-D on the morphology of MEL-85 cells. (**A**) Micrographs of control cells. (**B**) Micrographs of MEL-85 cells treated with 25 *μ*M MI-D. (**C**) Micrographs of MEL-85 cells treated with 50 *μ*M MI-D. MEL-85 cells were treated for 2 h, fixed and stained with Giemsa. Samples were observed using a bright-field microscope (Olympus BX40). Closed arrows point to cell shrinkage. Closed arrowheads show vacuolisation of cytoplasm. Open arrows indicate chromatin condensation. Open arrowheads indicate bleb formation in cell membranes (× 400).

shows micrographs of MEL-85 cells stained by Giemsa. It can be observed with treated cells (Figure 5B and C) that the presence of MI-D gave rise to a disruption of the interactions between cells and substratum. MI-D treated cells are not so spread out as control cells (Figure 5A). The results clearly demonstrate significant changes in cell shape, with cells becoming round when compared to those of the control, as was also observed in adhesion assays. The treatment with 25 *μ*M MI-D gave rise to shrinkage of some cells, presenting protrusions of the plasma membrane, which were pinched off to form membrane-enclosed similar apoptotic bodies probably with cytoplasmic and nuclear contents. Intense vacuolisation of cytoplasm was observed with treated cells. The concentration of 50 *μ*M affected the morphology of almost all of the cells. Condensed chromatin masses with intense eosinophilia and pyknotic nuclei were also observed with treated cells. Morphometric analysis permitted quantification of morphological changes and showed a reduction of 35% in the area of cells treated with 50 *μ*M MI-D. This concentration reduced cell elongation to 56% and increased cell roundness by 112%.

The article "Cytotoxic effect of a new 1,3,4-thiadiazolium mesoionic compound (MI-D) on cell lines of human melanoma" was published in 2004. Journal: Br J Cancer.

### Effect of MI-D on MEL-85 cytoskeleton organisation

In order to evaluate if the changes on cell shape were due to alterations on the actin organisation, an experiment using phalloidin-FITC conjugate was performed (Kusano *et al*, 2000). As can be observed in Figure 6

**Figure 6:** Effects of MI-D on F-actin cytoskeleton organisation of MEL-85 cells. (**A**) Micrographs of MEL-85 control cells (× 600). (**B**) MEL-85 control cells at a higher magnification showing details of well-organised F-actin cytoskeleton (× 1450). (**C**) Micrographs of MEL-85 cells treated with 50 *μ*M MI-D (× 600). (**D**) MEL-85 treated with 50 *μ*M MI-D, cells under a higher magnification, depicting disturbances to the organisation of F-actin molecules, concentrated at the edge of cells with a granular pattern (arrow) (× 1200). MEL-85 cells were treated with MI-D, fixed and labelled with a phalloidin-FITC conjugate and observed at a confocal fluorescence microscope (Confocal Radiance 2100, Bio-Rad) coupled to a Nikon Eclipse 800 with plan apochromatic objectives.

, organisation of actin cytoskeleton was completely disturbed by MI-D treatment. Fluorescence labelling of MEL-85 cells treated with MI-D did not give rise to the overall pattern that was observed in control cells, which showed a considerable organisation of F-actin fibres all over the cell body. MI-D treatment induced a reorganisation of the F-actin cytoskeleton architecture. Cells in the presence of MI-D did not spread and the filamentous structures disassembled or were reorganised to accumulate in the submembraneous area. Actin filaments turned into actin granules mainly localised on the edge of MEL-85 cells. These results point to a disruption of interactions between cells and the extracellular matrix.

The article "Cytotoxic effect of a new 1,3,4-thiadiazolium mesoionic compound (MI-D) on cell lines of human melanoma" was published in 2004. Journal: Br J Cancer.

## DISCUSSION

We are now able to show that MI-D has considerable cytotoxic and antiproliferative effects on human melanoma cell lines. These effects seem to be even more aggressive on human melanoma cells than those observed with B16-F10 murine melanoma cells (Senff-Ribeiro *et al*, 2003, 2004). For example, a dose of 10 *μ*M after 48 h incubation, on B16-F10 melanoma cells diminished their viability to ∼80% (Senff-Ribeiro *et al*, 2003, 2004) and in all the four human melanoma cell lines the viability was lower than 30% under these conditions. Interestingly, MI-D at a low concentration (5 *μ*M), gave rise to effects of a different magnitude on the viabilities of human melanoma cells. Under this condition, MEL-85 and MEWO cell lines (Figure 2A and D) were more sensitive to MI-D than SK-MEL and A2058 (Figure 2B and C). Inhibitions of different magnitude on the cell growth of different human melanoma cell lines were also observed. The concentration of 5 *μ*M allowed MEL-85 growth at a lower rate than that of the control (Figure 3A), but completely inhibited the growth of SK-MEL cells (Figure 3B). The results on viability and proliferation are compatible. As one can observe in Figures 2 and 3, MI-D was very cytotoxic to human melanoma cells and had also an antiproliferative effect. The antiproliferative effect of MI-D was present at both noncytotoxic and cytotoxic doses. The effects of MI-D on the viability and proliferation of the various human melanoma cell lines show MI-D to be a toxic drug for human melanoma cells.

Since tumour cell adhesion to ECM constituents is a fundamental step in tumour development and invasion (Mishima *et al*, 1998), we investigated the effect of MI-D on MEL-85 melanoma cells adhesion to laminin, fibronectin and matrigel. Low MI-D doses were used in order to minimise its extensive metabolic effects, so that the drug was used at subcytotoxic concentration to evaluate MEL-85 adhesion to ECM. Overall, 5 *μ*M MI-D caused a slight decrease of ∼5% on MEL-85 viability after 2 h. Under such an experimental condition, MI-D was able to inhibit cell adhesion when it was incubated with the cells for 2 h. Analysing the images of experiments (Figure 4D), we can observe that MI-D treatment promoted loss of cell spreading, which became round, suggesting a possible activity of MI-D on cytoskeleton organisation. These observations were confirmed by morphological and F-actin analyses. Loss of overall cell shape accompanied by cell shrinkage, membrane blebbing and chromatin condensation, besides disturbance of the cytoskeleton organisation, are often observed on apoptotic cells (Hengartner, 2000). The effects of MI-D on MEL-85 adhesion on ECM and morphology may be related to its cytotoxic activity. Although the four different cell lines showed slightly different sensitivities to MI-D, all of them responded to MI-D in a very similar way, so that the MEL-85 results on adhesion, morphology and cytoskeleton organisation probably represent an action of MI-D on human melanoma cell lines.

The article "Cytotoxic effect of a new 1,3,4-thiadiazolium mesoionic compound (MI-D) on cell lines of human melanoma" was published in 2004. Journal: Br J Cancer.

MI-D is an uncoupler of mitochondrial phosphorylation (Cadena *et al*, 1998), whose effects on membranes have been recognised (Cadena *et al*, 2002). Touching on this question, MI-D is an inhibitory uncoupler (Cadena *et al*, 1998) and according to Skulachev (1998) and others (Colombo *et al*, 2001), in some instances, an uncoupling action could explain the therapeutic effect of a drug. This seems true for the antitumour action of carbonylcyanide-*m*-chlorophenylhydrazone (CCCP) (Newell and Tannock, 1989) and other anticancer drugs (Keller *et al*, 1992). The induction of apoptosis could be a consequence of the cytotoxic activity of MI-D, as it is already known that drugs, which affect mitochondrial metabolism, might facilitate the induction of cell death and overcome apoptosis resistance in cancer cells (Susin *et al*, 1998; Colombo *et al*, 2001). Moreover, since membrane proteins are highly dependent on membrane organisation and fluidity (Lopez and Kosk-Kosika, 1997), the effects of MI-D on membranes could disturb recognition sites, which are necessary for adhesion.

In conclusion, MI-D is a potent drug against human melanoma cells and this is the first study on its effects against these cells, as well as for a mesoionic compound of the 1,3,4-thiadiazolium class. Besides its cytotoxic properties, MI-D also interferes in cell features involved in tumour development, such as adhesion to ECM components. These results, combined with previous data (Senff-Ribeiro *et al*, 2003, 2004) that showed MI-D to be a potent drug against B16-F10 murine melanoma both *in vitro* and *in vivo*, emphasise that MI-D could be a promising drug for the treatment and study of melanoma.

## References

[bib1] Badachikar SV, Tikare RK, Puranik GS (1986) Synthesis, reactions and biological activity of 3-[*p*-(*N*-methyl/ethyl-*N*-phenylcarbamoyl)] phenylsydnones. Indian J Chem 25B: 1079–1080

The article "Cytotoxic effect of a new 1,3,4-thiadiazolium mesoionic compound (MI-D) on cell lines of human melanoma" was published in 2004. Journal: Br J Cancer.

[bib2] Cadena SMSC, Carnieri EGS, Echevarria A, Oliveira MBM (1998) Effect of MI-D, a new mesoionic compound, on energy-linked functions of rat liver mitochondria. FEBS Lett 440: 46–50986242210.1016/s0014-5793(98)01427-6

[bib3] Cadena SMSC, Carnieri EGS, Echevarria A, Oliveira MBM (2002) Interference of MI-D, a new mesoionic compound, on artificial and native membranes. Cell Biochem Funct 20: 31–371183526810.1002/cbf.932

[bib4] Cheung KK, Echevarria A, Galembeck S, Maciel MAM, Miller J, Rumjanek VM, Simas AM (1992) Mesoionic compounds 3. Structure of the hydrochloride of 5-(4-methoxyphenyl)-1,3,4-thiadiazolium-2-phenylamine. Acta Crystallogr 48: 1471–1474

[bib5] Colombo P, Gunnarsson K, Iatroupoulos M, Brughera M (2001) Toxicological testing of cytotoxic drugs (Review). Int J Oncol 19: 1021–10281160500410.3892/ijo.19.5.1021

[bib6] Corell T, Pedersen SB, Lissau B, Moilanen E, Mëtsa-Ketelä T, Kankaanranta H, Vuorinen P, Vapaatalo H, Rydell E, Andersson R, Marcinkiewicz E, Korbut R, Gryglewski RJ (1994) Pharmacology of mesoionic oxatriazole derivatives in blood, cardiovascular and respiratory systems. Pol J Pharmacol 46: 553–5667542520

[bib7] Engvall E, Ruoslahti E (1977) Binding of soluble form of fibroblast surface protein, fibronectin, to collagen. Int J Cancer 20: 1–590317910.1002/ijc.2910200102

[bib8] Grynberg N, Gomes R, Shinzato T, Echevarria A, Miller J (1992) Some new aryl sydnones: effects on murine tumors. Anticancer Res 12: 1025–10281320354

[bib9] Grynberg N, Santos AC, Echevarria A (1997) Synthesis and *in vivo* antitumor activity of new heterocycles derivatives of 1,3,4-thiadiazolium-2-aminide class. Anti-Cancer Drugs 8: 88–91914761710.1097/00001813-199701000-00012

[bib10] Hengartner MO (2000) The biochemistry of apoptosis. Nature 407: 770–7761104872710.1038/35037710

[bib11] Hogg N, Darley-Usmar VM, Wilson MT, Moncada S (1992) Production of hydroxyl radicals from simultaneous generation of superoxide and nitric oxide. Biochem J 281: 419–424131059510.1042/bj2810419PMC1130701

[bib12] Kankaanranta H, Rydell E, Peterson AS, Holm P, Moilanen E, Corell T, Karup G, Vuorinen P, Pedersen SB, Wennmalm A, MetsaKeleta T (1996) Nitric oxide-donating properties of mesoionic 3-aryl substituted oxatriazole-5-imine derivatives. Br J Pharmacol 117: 401–406882152610.1111/j.1476-5381.1996.tb15204.xPMC1909319

[bib13] Keller BJ, Marsman DS, Popp JA, Thurman RG (1992) Several nongenotoxic carcinogens uncouple mitochondrial oxidative phosphorylation. Biochim Biophys Acta 1102: 237–244139082510.1016/0005-2728(92)90105-b

The article "Cytotoxic effect of a new 1,3,4-thiadiazolium mesoionic compound (MI-D) on cell lines of human melanoma" was published in 2004. Journal: Br J Cancer.

[bib14] Kier LB, Roche EB (1967) Medicinal chemistry of the mesoionic compounds. J Pharm Sci 56: 148–16910.1002/jps.26005602025338256

[bib15] Kleinman HK, McGarvey ML, Hassel JR, Star VL, Cannon FB, Laurie GW, Martin GR (1986) Basement membrane complexes with biological activity. Biochemistry 25(2): 312–318293744710.1021/bi00350a005

[bib16] Kusano Y, Oguri K, Nagayasu Y, Munesue S, Ishihara M, Saiki I, Yonekura H, Yamamoto H, Okayama M (2000) Participation of syndecan 2 in the induction of stress fiber formation in cooperation with integrin *α*5*β*1: Structural characteristics of heparan sulfate chains with avidity to COOH-terminal heparin-binding domain of fibronectin. Exp Cell Res 256: 434–4441077281610.1006/excr.2000.4802

[bib17] Lopez MM, Kosk-Kosika P (1997) Entropy-driven interactions of anesthetics with membrane proteins. Biochemistry 36: 8864–8872922097310.1021/bi970028w

[bib18] Majid PA, DeFeyter PJF, Van der Wall EE, Wardeh R, Ross JP (1980) Molsidomine in the treatment of patients with angina pectoris. N Engl J Med 302: 1–6698569710.1056/NEJM198001033020101

[bib19] Mishima T, Murata J, Toyoshima M, Fujii H, Nakajima M, Hayashi T, Kato T, Saiki I (1998) Inhibition of tumor invasion and metastasis by calcium spirulan (Ca-SP), a novel sulfated polysaccharide derived from blue-green alga, *Spirulina platensis*. Clin Exp Metast 16: 541–55010.1023/a:10065943186339872601

[bib20] Montanari CA, Beezer AE, Sandall JPB, Montanari MLC, Miller J, Giesbrecht AM (1992) On the interaction of some mesoionic compounds with *Saccharomyces cerevisiae* by biological microcalorimetry. Rev Microbiol 23: 274–278

[bib21] Mosmann T (1983) Rapid colorimetric assay for cellular growth and survival: application to proliferation and cytotoxicity assays. J Immunol Methods 65: 55–63660668210.1016/0022-1759(83)90303-4

[bib22] Moustafa MAA, Eisa HM (1991) Synthesis and antimicrobial activity of 3-(substituted–phenyl)–sydnones. Arch Pharmacol 325: 397–40110.1002/ardp.199232507061417454

[bib23] Newell KJ, Tannock IF (1989) Reduction of intracellular pH as a possible mechanism for killing cells in acidic regions of solid tumors: effects of carbonylcyanide-3-chlorophenylhydrazone. Cancer Res 49: 4477–44822743336

[bib24] Newton CG, Ramsden CA (1982) Meso-ionic heterocycles. Tetrahedron 38: 2965–3011

[bib25] Ollis WD, Ramsden CA (1976) Meso-ionic compounds. Adv Heterocycl Chem 19: 1–121

[bib26] Paulsson M, Aumailley M, Deutzmann R, Timpl R, Beck R (1987) Laminin–nidogen complex: extraction with chelating agents and structural characterization. Eur J Biochem 166: 11–19310991010.1111/j.1432-1033.1987.tb13476.x

[bib27] Phillips HJ (1973) Dye exclusions tests for cell viability. In Tissue Culture, Methods and Applications, Kruse JR, Patterson JRMK (eds) pp 406–408, New York: Academic Press

The article "Cytotoxic effect of a new 1,3,4-thiadiazolium mesoionic compound (MI-D) on cell lines of human melanoma" was published in 2004. Journal: Br J Cancer.

[bib28] Rehse K, Ciborski T, Müller B (1995) Platelet aggregation inhibiting and anticoagulant effects of oligoamines. XXVII: inhibition of leucocyte adherence to endothelium by oligoamine RE 1492C and the NO-donor RE 2047. Arch Pharm (Weinheim) 328: 125–126772673610.1002/ardp.19953280206

[bib29] Rehse K, Konig P (1995) New NO-donors with antithrombotic and vasodilating activities. XII. Mesoionic oxatriazoles and related monocyclic nitrosohydrazine derivatives. Arch Pharmacol 328: 137–14210.1002/ardp.199532802097726739

[bib30] Rudolph W, Derschinger J (1991) Clinical comparison of nitrates and sydnonimines. Eur Heart J 12: 33–4110.1093/eurheartj/12.suppl_e.331790782

[bib31] Saiki I, Iida J, Murata J, Ogawa R, Nishi N, Sugimura K, Tokura S, Azuma I (1989) Inhibition of the metastasis of murine malignant melanoma by synthetic polymeric peptides containing core sequences of cell-adhesive molecules. Cancer Res 49: 3815–38222736523

[bib32] Satyanarayana K, Rao MNA (1995) Synthesis and anti-inflammatory, analgesics and antipyretic testing of 4-[1-oxo-(3-substituted aryl)-2-propenyl]-3-phenylsydnones and of 3-[4-[3-(substituted aryl)-1-oxo-2-propenyl] phenyl] sydnones. J Pharmacol Sci 84: 263–26610.1002/jps.26008402287738813

[bib33] Senff-Ribeiro A, Echevarria A, Silva EF, Veiga SS, Oliveira MBM (2003) Effect of a new 1,3,4-thiadiazolium mesoionic compound (MI-D) on B16-F10 murine melanoma. Melanoma Res 13(5): 465–4721451278810.1097/00008390-200310000-00005

[bib34] Senff-Ribeiro A, Echevarria A, Silva EF, Veiga SS, Oliveira MBM (2004) Antimelanoma activity of 1,3,4-thiadiazolium mesoionics: a structure–activity relationship study. Anti-Cancer Drugs 15(3): 269–2751501436110.1097/00001813-200403000-00012

[bib35] Shinzato TO, Grynberg N, Gomes RM, Echevarria A, Miller J (1989) Antitumor activity of new mesoionic compounds against three murine tumors. Med Sci Res 17: 865–866

[bib36] Skulachev VP (1998) Uncoupling: new approaches to an old problem of bioenergetics. Biochim Biophys Acta 1363: 100–124950707810.1016/s0005-2728(97)00091-1

[bib37] Susin SA, Zamzami N, Kroemer G (1998) Mitochondria as regulators of apoptosis: doubt no more. Biochim Biophys Acta 1366: 151–165971478310.1016/s0005-2728(98)00110-8

